The article "Effective Analysis of Multichannel Functional Electrical Stimulation plus Early Rehabilitation Training for Hemiplegic Patients after Stroke" was retracted in 2023. Reasons: suspected computer-generated content; unreliable results or conclusions; concerns about the data; concerns about the results or conclusions.

# Effective Analysis of Multichannel Functional Electrical Stimulation plus Early Rehabilitation Training for Hemiplegic Patients after Stroke

**DOI:** 10.1155/2022/6061652

**Published:** 2022-07-07

**Authors:** Yan Hou, Li Yang

**Affiliations:** Department of Internal Medicine, No. 215 Hospital of Shaanxi Nuclear Industry, Xianyang, Shaanxi Province, China

## Abstract

**Purpose:**

The research paper aims to investigate the value of multichannel functional electrical stimulation (FES) plus early rehabilitation training for hemiplegic patients after stroke attacks and assesses the impact of the combined therapy on walking capacity and daily life activities of patients.

**Methods:**

Totally, 100 hemiplegic patients after stroke treated in No. 215 Hospital of Shaanxi Nuclear Industry from March 2019 to July 2020 were recruited and randomized into the control group and study group, with 50 cases in each group. The control group received early rehabilitation training, and the study group received multiple channel FES plus early rehabilitation. The rehabilitation effective rate, the Fugl–Meyer Assessment (FMA), the Berg Balance Scale (BBS), National Institutes of Health Stroke Scale (NIHSS), Barthel index (BI), the Quality of Life index (QLI), Mental Status Scale in Nonpsychiatric Settings (MSSNS), Self-rating Anxiety Scale (SAS), Self-rating depression scale (SDS), and the incidence of adverse response were evaluated.

**Results:**

The study group patients had higher scores in FMA, BBS, BI, and QLI than the control group. Multiple channel FES plus early rehabilitation adopted in the study group resulted in a higher rehabilitation efficacy and a longer walking duration at 1, 2, and 4 weeks after the treatment. NIHSS score, MSSNS score, SAS score, SDS score, and incidence rate of adverse response in the study group were significantly lower compared to those of the control group.

**Conclusions:**

Multichannel FES plus early rehabilitation training effectively enhances the rehabilitation of patients after stroke attacks.

## 1. Introduction

Stroke is mostly caused by brain hypoxia due to the insufficient supply of blood to the brain after the rupture of atherosclerotic plaque [1]. Stroke is subdivided into multiple types such as ischemic, hemorrhagic, and transient ischemic stroke, and the treatment method for each type varies significantly [2, 3]. The main symptoms of strokes include paralysis, limb numbness, language impairment, memory dysfunction, delayed response, seizures, and even coma, and death may occur after cerebral hemorrhage [4]. Thus, early interventions for stroke are conducive to the prevention of permanent brain damage and complications [5]. In traditional Chinese medicine (TCM), rehabilitation care after stroke attacks focuses on the elimination of evil qi and the restoration of healthy qi in the patient's body [6]. TCM rehabilitation nursing improves patient treatment compliance, restoring the limb function of patients and lowering the disability rate through psychological and physical interventions such as psychological management, acupoint massage, and health education [7]. Limited mobility, or reduced walking capacity, is one of the sequelae of stroke and is frequently observed in most stroke survivors [8], and it is the result of improper management of the paralyzed lower limb muscles. In general, thrombolytic therapy performed within 2 hours after stroke attacks substantially lowers the risk of sequelae. However, it has been reported that timely and effective thrombolytic management is absent in most stroke cases, resulting in compromised quality of life of patients [9]. Electrical stimulation rehabilitation training is commonly used in the rehabilitation of hemiplegic patients, with high efficiency and low risks. It has been reported that functional electrical stimulation (FES) plus early rehabilitation training had a favorable application effect in the rehabilitation of patients with cerebral infarction [10]. The multichannel FES is a type of rehabilitation that induces afferent input and muscle contractions to perform rehabilitation training. It facilitates the rehabilitation process of the patient and contributes significantly to the correction of gait asymmetries [11]. The present study was conducted to explore the effects of multichannel FES combined with early rehabilitation training in patients after stroke attacks and analyze the impact of the combined therapy on their walking capacity and quality of life.

## 2. Materials and Methods

### 2.1. General Information

In this retrospective study, a total of 100 hemiplegic admitted patients after stroke attacks treated in No. 215 Hospital of Shaanxi Nuclear Industry from March 2019 to July 2020 were recruited and assigned to a control group and study group, with 50 cases in each group. This study was approved by the ethical committee of the No. 215 Hospital of Shaanxi Nuclear Industry (approval no. 2018-223/241). All patients voluntarily participated in the study after being fully informed about the details of the research and signed the informed consent document.

### 2.2. Inclusion and Exclusion Criteria

#### 2.2.1. Inclusion Criteria

Inclusion criteria were as follows: (1) patients who met the clinical manifestations of stroke hemiplegia; (2) patients aged between 18 and 80 years; (3) patients without other organic diseases; and (4) patients without a history of drug addiction were included.

#### 2.2.2. Exclusion Criteria

Exclusion criteria were as follows: (1) patients with hemiplegia; (2) patients without no cerebral infarction; (3) patients with unconsciousness; and (4) patients with liver and kidney problems were excluded.

### 2.3. Methods

The control group patients received early rehabilitation training, including walking exercises, flexibility exercises, acupuncture, and TCM massage. Bedridden patients were assisted to turn over to avoid pressure sores.

The patients in the study group received additional multichannel FES plus early rehabilitation training. The early rehabilitation training protocol was identical to that given to the patients in the control group. During the FES therapy, the electrodes of the electrical stimulator were placed at the location of the extensor, gastrocnemius, and biceps femoris muscles and energized. The stimulation frequency was set at 30 Hz and appropriately adjusted according to patients' tolerance. The patients received FES therapy for 30 minutes daily, and the duration of FES therapy was 2 weeks.

### 2.4. Observation of Indexes

#### 2.4.1. Rehabilitation Efficiency

The efficiency was considered significantly effective if the limb motor function and walking capability of the patients is substantially restored without adverse effects. The efficiency was considered effective if the limb motor function and walking capability of the patients is partially restored, and they could walk under assistance. The efficiency was considered ineffective if no restoration of the limb motor function and walking capability of the patients was observed.

#### 2.4.2. Fugl–Meyer Assessment (FMA)

The full score of FMA is 100 points, with 66 points for the assessment of upper limb function and 34 points for the lower limb function. A higher score indicates better motor function [12].

#### 2.4.3. Berg Balance Scale (BBS)

The full score of BBS is 56 points. A higher score indicates better balance ability [13].

#### 2.4.4. National Institutes of Health Stroke Scale (NIHSS)

The NIHSS neurological score ranges between 0 and 42 points. A higher score indicates a more severe neurological deficit. If the score is 0 or 1, it indicates a normal condition. A score between 1 to 4 points indicates mild stroke. A score between 5 to 15 points indicates moderate stroke. A score between 16 to 20 points indicates moderately severe stroke, and a score between 21 to 42 points indicates severe stroke [14].

#### 2.4.5. Barthel Index (BI)

The BI index has 100 points. A score of 100 points indicates no dependency on external assistance for daily living, 61–99 points suggests moderate dependency, 41–60 points indicates severe dependency, and less than 40 points indicates total dependency [15].

The QLI scale has a full score of 10 points. The higher the score, the better the quality of life [16].

#### 2.4.6. Mental Status Scale in Nonpsychiatric Settings (MSSNS)

The MSSNS score has a total score of 100 points. A score less than 60 points suggests normal psychological status, a score between 60 to 70 points indicates mildly abnormal psychological status, and a score more than 70 points indicates abnormal psychological status [17].

#### 2.4.7. Self-Rating Anxiety Scale (SAS) and Self-Rating Depression Scale (SDS)

The SAS has a total score of 50 points. A score less than 50 indicates normal status, a score between 50 and 59 indicate mild anxiety, a score between 60 and 69 indicate moderate anxiety, and a score more than 70 indicates severe anxiety. The SDS has a score of 53 points for reference value. A score less than 53 points indicate normal status, a score between 53 and 62 indicate mild depression, a score between 63 and 72 indicate moderate depression, and a score more than 72 points indicate severe depression [18].

### 2.5. Statistics

SPSS 20.0 software was used for data analyses, and GraphPad Prism 7 (GraphPad Software, San Diego, USA) was used to plot the graphs. Measurement data are represented as mean ± standard deviation and analyzed using the *t*-test. Enumeration data are represented as *n* (%) and analyzed using the chi-square test. *P* < 0.05 indicated a statistically significant difference.

## 3. Results

### 3.1. Comparison of the General Data

Patients in the control group were aged between 43 and 72 years, and those in the study group were aged between 45 and 73 years. There were no significant differences in the baseline characteristics between the two groups of patients (*P* > 0.05), as shown in Table 1.

### 3.2. Comparison of Rehabilitation Efficiency

The rehabilitation efficiency of the study group was significantly higher than that of the control group (*P* < 0.05), as shown in Table 2.

### 3.3. Comparison of FMA Score and BBS Score

The study group had significantly higher FMA and BBS scores than the control group, as shown in Figure 1.

### 3.4. Comparison of NIHSS Score and BI

The study group showed significantly lower NIHSS scores and higher BI scores than the control group, as shown in Figure 2.

### 3.5. Comparison of QLI Score and MSSNS Score

The patients in the study group had higher QLI scores and lower MSSNS scores compared to the control group (*P* < 0.05), as shown in Table 3.

### 3.6. Comparisons of SAS Score and SDS Score

The SAS and SDS scores in the study group were lower than those of the control group, as shown in Figure 3.

### 3.7. Comparison of the Incidence of Adverse Response

Adverse responses that occurred during treatment mainly included urinary retention, bedsore, and respiratory system infection. The incidence of adverse responses in the study group was lower than in the control group (*P* < 0.05), as shown in Table 4.

### 3.8. Comparison of Walking Capacity Restoration

Patients in the study group could achieve longer walking duration than those in the control group at 1, 2, and 4 weeks after treatment (*P* < 0.05), as shown in Figure 4.

## 4. Discussion

Stroke is a life-threatening disease with a high prevalence in the elderly population. Manifestations of stroke mainly include motor deficit and memory dysfunction, which significantly compromise the quality of life of patients [19]. Hemiplegia is one of the common sequelae of stroke, which manifests as unilateral limb stiffness, weakness, and movement disorders, resulting in abnormal gait [20]. Currently, effective treatment for hemiplegic patients is timely rehabilitation training to restore balance and walking capacity. Multichannel FES therapy is designed to promote target movement by neurological stimulation [21].

The results of the present study showed that the patients in the study group receiving multichannel FES plus early rehabilitation training had higher FMA, BBS, BI, and QLI scores, higher rehabilitation efficiency, and a better walking capacity at 1, 2, and 4 weeks after treatment (*P* < 0.05), suggesting that multichannel FES plus early rehabilitation training could significantly improve the limb motor of patients, thereby improving their living ability. In rehabilitation, the evaluation of motor function and quality of life contributes to the timely adjustment of treatment plans and enhancement of the overall rehabilitation outcomes [22]. The NIHSS score, MSSNS score, SAS score, SDS score, and incidence of adverse response in the study group were significantly lower than those in the control group (*P* < 0.05), indicating that the combined therapy of early rehabilitation training and multichannel FES achieved the better restoration of neurological functions and improvement of psychological status.

## 5. Conclusion

Multichannel FES plus early rehabilitation training for hemiplegic patients after stroke attacks significantly improves the rehabilitation training effect, accelerates the recovery, and boosts the quality of life of the patients.

## Figures and Tables

**Figure 1:** Comparison of FMA score and BBS score. ^*∗∗∗*^*P* < 0.001.

**Figure 2:** Comparison of NIHSS score and BI. ^*∗∗∗*^*P* < 0.001.

**Figure 3:** SAS and SDS score. ^*∗∗∗*^*P* < 0.001.

**Figure 4:** Comparison of the duration of one-time walking training 1 week, 2 weeks, and 4 weeks after treatment. ^*∗∗∗*^*P* < 0.001.

**Table 1:** General information.

Group		Study group (*n* = 50)	Control group (*n* = 50)	*t*/*χ*2	*P*
Gender (male/female)		26/24	24/26	0.16	0.69
Age ($\bar{x}$ ± *s*, years)		60.58 ± 7.33	60.00 ± 7.67	0.39	0.70
Height ($\bar{x}$ ± *s*, cm)		163.21 ± 8.52	163.38 ± 8.60	0.10	0.92
Weight ($\bar{x}$ ± *s*, kg)		61.05 ± 6.47	61.39 ± 6.29	0.27	0.79
Medical history ($\bar{x}$ ± *s*, months)		1.38 ± 0.75	1.39 ± 0.70	0.07	0.95
Alcohol history ($\bar{x}$ ± *s*, years)		10.92 ± 2.80	10.55 ± 2.94	0.64	0.52
Epilepsy	Left (*n*)	30	33	0.39	0.53
	Right (*n*)	20	17		
Hypertension (*n*)		11	12	0.06	0.81
Diabetes (*n*)		17	18	0.04	0.83
Hyperlipidemia (*n*)		20	19	0.04	0.84

**Table 2:** Comparison of rehabilitation effective rate (*n*, %).

	Significantly effective	Effective	Ineffective	Overall response rate
Study group (*n* = 50)	32	13	5	45 (90.00)
Control group (*n* = 50)	19	14	17	33 (66.00%)
*χ*2				8.39
*P*				<0.001

**Table 3:** QLI and MSSNS score ($\bar{x}$ ± *s*).

	QLI score	MSSNS score
Study group (*n* = 50)	55.33 ± 4.61	39.67 ± 2.05
Control group (*n* = 50)	47.71 ± 3.81	44.57 ± 2.31
*t*	9.01	11.22
*P*	<0.001	<0.001

**Table 4:** Comparison of the incidence of adverse response (*n*, %).

	Urinary retention	Bedsore	Respiratory system infection	Adverse response rate
Study group (*n* = 50)	2	4	1	7 (14.00)
Control group (*n* = 50)	6	8	2	16 (32.00)
*χ*2				4.57
*P*				0.03

## Data Availability

All data generated or analyzed during this study are included within the published article.
